The article "Human cathelicidin LL-37 enhance the antibiofilm effect of EGCG on Streptococcus mutans" was retracted in 2017. Reasons: copyright claims; concerns about the data.

# Human cathelicidin LL-37 enhance the antibiofilm effect of EGCG on *Streptococcus mutans*

**DOI:** 10.1186/s12903-016-0292-y

**Published:** 2016-09-22

**Authors:** Yi-jie Guo, Bo Zhang, Xue-song Feng, Hui-xun Ren, Ji-ru Xu

**Affiliations:** 1 Department of Pathogenic Microbiology and Immunology, School of Basic Medical Sciences, Xi’an Jiaotong University, Yanta West Road No.76, Xi’an, 710061 ShaanXi China; 2 Clinical Laboratory, AnKang City Central Hospital, Jinzhou South Road No.85, AnKang, 725000 ShaanXi China; 3 Key Laboratory of Environment and Genes Related to Diseases, Ministry of Education of China, Xi’an Jiaotong University, Yanta West Road No.76, Xi’an, 710061 ShaanXi China

**Keywords:** LL-37, EGCG, *Streptococcus mutans*, Biofilm

## Abstract

**Background:**

*Streptococcus mutans* forms biofilms as a resistance mechanism against antimicrobial agents in the human oral cavity. We recently showed that human cathelicidin LL-37 exhibits inhibitory effects on biofilm formation of *S. mutans* through interaction with lipoteichoic acid (LTA), but without antibacterial or biofilm dispersal abilities. (−)-Epigallocatechin gallate (EGCG) is the most abundant constituent of tea catechins that has the greatest anti-infective potential to inhibit the growth of various microorganisms and biofilm formation. Therefore, in this study, we evaluated whether LL-37 interacts with EGCG to enhance the antibiofilm effect of EGCG on *S. mutans* biofilm formation.

**Methods:**

Clinical *S. mutans* strains (*n* = 10) isolated from children’s saliva were tested in a biofilm formation assay. The antibiofilm effect of EGCG with and without LL-37 was analyzed by the minimum biofilm eradication concentration assay and confirmed using field emission-scanning electron microscopy. In addition, the interaction among EGCG, LL-37, and LTA of *S. mutans* was determined using quartz crystal microbalance analysis.

**Results:**

EGCG killed 100 % of planktonic *S. mutans* within 5 h, inhibited biofilm formation within 24 h, and reduced bacteria cells in preformed biofilms within 3 h at a concentration of 0.2 mg/mL. However, EGCG did not appear to interact with LTA. LL-37 effectively enhanced the bactericidal activity of EGCG against biofilm formation and preformed biofilms as determined by quantitative crystal violet staining and field emission-scanning electron microscopy. In addition, quartz crystal microbalance analysis revealed that LL-37 interacted with EGCG and promoted binding between EGCG and LTA of *S. mutans*.

**Conclusions:**

We show that LL-37 enhances the antibiofilm effect of EGCG on *S. mutans*. This finding provides new knowledge for dental treatment by using LL-37 as a potential antibiofilm compound.

The article "Human cathelicidin LL-37 enhance the antibiofilm effect of EGCG on Streptococcus mutans" was retracted in 2017. Reasons: copyright claims; concerns about the data.

**Electronic supplementary material:**

The online version of this article (doi:10.1186/s12903-016-0292-y) contains supplementary material, which is available to authorized users.

## Background

Pathogenic bacteria can form biofilms that cause much infectious disease in the human oral cavity. Among these diseases, dental caries is one of the most ubiquitous biofilm-dependent oral diseases worldwide, which frequently occurs in both children and adults [1]. Oral streptococci, including *Streptococcus mutans* and *Streptococcus sobrinus*, are generally considered the primary etiologic agents of dental caries [2, 3]. One of the most well-documented virulence characteristics of *S. mutans* is its ability to establish cariogenic biofilms on tooth surfaces as an assembled extracellular matrix [4, 5]. Extracellular polymeric substances, especially water-insoluble glucans, are the main constituents of the matrix and can mediate *S. mutans* adherence [6, 7]. Other constituents such as extracellular DNA [8] and lipoteichoic acids (LTA) have also been found in high concentrations in the matrix of cariogenic biofilms [9, 10].

Tea is the most frequently consumed beverage in the world after water [11]. The antimicrobial activity of tea was first demonstrated almost 100 years ago by McNaught [12]. Green tea (*Camellia sinensis*) is a non-fermented tea that has more beneficial effects than black tea or oolong tea [13]. It has been observed that catechin components of green tea are responsible for its antibacterial activity, and (−)-epicatechin gallate, (−)-epigallocatechin (EGC), and (−)-epigallocatechin gallate (EGCG) constitute the most important antibacterial agents of tea catechins [14, 15].

EGCG is the most abundant constituent of tea catechins that has the greatest anti-infective ability by inhibiting the growth of various microorganisms [16], biofilm formation [17], and quorum sensing [18, 19]. Xu et al. reported that EGCG inhibits the growth of *S. mutans*, decreases glucosyltransferases activity, and suppresses *gtf* genes, which are associated with bacterial biofilm formation [20, 21]. However, the effects of EGCG on biofilm and cariogenic virulence factors of oral streptococci other than glucosyltransferases have not been well documented, especially regarding its potential interaction with LTA.

The antibacterial peptide LL-37 is the only member of the cathelicidin family found in humans. LL-37 is an 18-kDa peptide [22] with 37 amino acid residues that start with two leucines [23]. LL-37 is expressed in many tissues and body fluids, such as saliva, gingiva, sweat, amniotic fluids, and seminal plasma [24]. It has been reported that the intravital concentration of LL-37 is about 86 μg/mL in seminal plasma of healthy donors [25], and ranges from less than 1.2 to more than 80 μg/mL in unstimulated and nonpurulent nasal secretions [26], respectively. Cariogenic species, such as *S. sobrinus*, *Lactobacillus paracasei*, and *Actinomyces viscosus* have been reported to be resistant to LL-37 through growth inhibition and bactericidal tests [27], especially when biofilm formation occurred. We recently showed that LL-37 has the ability to bind to LTA of *S. mutans*, inhibiting biofilm formation [28]. Therefore, in this study, we evaluated whether LL-37 could be used as a binding agent to enhance the interaction between EGCG and LTA of *S. mutans* to increase the antibiofilm effect of EGCG.

The article "Human cathelicidin LL-37 enhance the antibiofilm effect of EGCG on Streptococcus mutans" was retracted in 2017. Reasons: copyright claims; concerns about the data.

## Methods

### Bacterial strains and culture conditions

Ten clinical *S. mutans* strains isolated from children’s saliva were kindly provided by Dr. E. Isogai [29]. Bacteria were grown in brain heart infusion (BHI) broth (Merck KGaA, Darmstadt, Germany) for 24 h at 37 °C. The present study was approved by the Ethics Committee of Xi’an Jiaotong University Faculty of Medicine (XJTU2014-014).

### Catechin and antimicrobial peptide

EGCG (NH020403) was purchased from Nagara Science Co. Ltd. (Gifu, Japan). EGCG was dissolved in absolute ethyl alcohol at a concentration of 10 mg/mL. Then, EGCG/ethanol was used a concentration of 2 % to yield a maximum concentration of 0.2 mg/mL. LL-37 (sequence: LLGDF FRKSK EKIGK EFKRI VQRIK DFLRN LVPRT ES) powder was synthesized as described previously using the solid-phase method [30]. Briefly, the peptide was purified (>99.9 %) by reverse-phase high-performance liquid chromatography (Model LC-8A; Shimadzu Corporation, Kyoto, Japan) on a YMC-A 302 column (YMC Co. Ltd., Kyoto, Japan). The final product was confirmed by electrospray ionization mass spectrometry and conserved by suspension in Hank’s balanced salt solution (HBSS, pH 7.4; Gibco, Grand Island, NY, USA).

### Growth inhibition test

Precultured bacteria were measured at an optical density (OD) of 660 nm using an ultraviolet/visible spectrophotometer (Ubest-35; JASCO Corporation, Tokyo, Japan). Samples were adjusted to OD_660_ = 0.5 using BHI broth. Then, bacteria were diluted to a final concentration of 10^3^–10^4^ Colony-forming unit (CFU)/mL with BHI broth, and 1 mL of adjusted culture and 1 mL of EGCG solution were mixed together [28, 31]. The EGCG solution was prepared by two-fold serial dilution in BHI broth. Each mixture solution was incubated at 37 °C. The bactericidal activity of EGCG was estimated by measuring the minimum inhibitory concentration (MIC) and minimum bactericidal concentration (MBC) at 3, 5, and 24 h of incubation according to Clinical and Laboratory Standards Institute 2014 (CLSI) guidelines. After each incubation, 100 μL of EGCG–cell suspension was removed and inoculated on BHI agar plates. The plates were incubated for 48 h at 37 °C, followed by colony counting (CFU/mL). Control samples were prepared by mixing 1 mL of bacterial suspension with 0.9 mL of BHI broth and 0.1 mL of HBSS. The MIC was defined as the lowest concentration of EGCG that inhibited visible bacterial growth after overnight incubation. The MBC was defined as the lowest concentration of EGCG that killed 99.9 % of the initial inoculum.

The article "Human cathelicidin LL-37 enhance the antibiofilm effect of EGCG on Streptococcus mutans" was retracted in 2017. Reasons: copyright claims; concerns about the data.

### Biofilm formation assays

Biofilm formation was measured under two static conditions using a quantitative crystal violet assay on a polystyrene 96-well, minimum biofilm eradication concentration plate (MBEC; Biosurface Technologies, Bozeman, MT, USA) as described previously [32]. The MBEC biofilm assay used 96 polystyrene pegs that fit the wells of a conventional plate. Briefly, overnight cultures of S. mutans were diluted to OD_660_ = 0.5 (1 × 10^7^ CFU/mL) in fresh BHI. Two hundred microliters of bacterial suspensions were transferred to a 96-well microtiter plate with 20 μL of varying concentrations of EGCG in the presence or absence of LL-37 (final concentration of 80 μL/mL). The microtiter plates were then incubated at 37 °C with shaking for 12, 24, and 36 h. After incubation, the pegs were washed several times with phosphate buffered solution (PBS) and then fixed with 200 μL of 100 % ethanol prior to staining for 2 min with 200 μL of 0.41 % (wt/vol) crystal violet in 12 % ethanol (Bio Chemical Sciences, Swedesboro, NJ, USA). The pegs were washed several times with PBS to remove excess stain. Quantitative assessment of biofilm formation was performed by the immersion of pegs in a sterile microtiter plate containing 200 μL of 100 % ethanol and incubation at room temperature for 10 min. The absorbance at 550 nm was then determined. Three independent experiments were performed for each abovementioned assay.

### Biofilm susceptibility assays

To measure the antimicrobial susceptibility of *S. mutans* growing in biofilms, the MBEC High-throughput (HTP) Assay (Innovotech Inc., Edmonton, Alberta, Canada) was performed [33]. Briefly, overnight cultures of *S. mutans* were diluted to OD_660_ = 0.5 (1 × 10^7^ CFU/mL) in fresh BHI. Then, 200 μL of bacterial suspensions was transferred to the wells of a MBEC microtiter plate and the MBEC lid was placed on top of the wells. Biofilms were grown on the MBEC pegs at 37 °C under shaking conditions for 24 h. The lid was removed and transferred to a new plate with wells filled with varying concentrations of EGCG in the presence or absence of LL-37 (final concentration of 80 μL/mL), and incubated for 3 and 5 h at 37 °C. After each incubation, the lid was gently washed twice with 200 μL of PBS to remove non-adherent cells. Adherent biofilms were fixed with 200 μL of 100 % ethanol prior to staining for 2 min with 200 μL of 0.41 % (wt/vol) crystal violet in 12 % ethanol. The pegs were washed several times with PBS to remove excess stain. Quantitative assessment of biofilm formation was performed by the immersion of pegs in a sterile polystyrene microtiter plate which contained 200 μL of 100 % ethanol. The plate was incubated at room temperature for 10 min, then the absorbance at 550 nm was determined using a microplate spectrophotometer. Three independent experiments were performed for each assay.

The article "Human cathelicidin LL-37 enhance the antibiofilm effect of EGCG on Streptococcus mutans" was retracted in 2017. Reasons: copyright claims; concerns about the data.

### Field emission-scanning electron microscopy (FE-SEM)

To visualize the effects of EGCG on planktonic bacteria [28, 31], 10 μL of EGCG solution (0.2 mg/mL) was plated on a glass slide followed by 10 μL of bacteria mixed with the solution. This cell suspension was then incubated at 37 °C for 24 h and dried. Saturated 70 % ethanol was then applied for 5 min, followed by saturated 100 % ethanol for 5 min, and then the sample was dried. The sample was then coated with palladium alloy and examined using FE-SEM (SU8000; Hitachi High-Technologies Corporation, Tokyo, Japan).

To visualize the effect of EGCG on biofilms, the MBEC HTP Assay (Innovotech Inc.) was used [28]. Pegs with adherent biofilms were removed from the MBEC biofilm assay and rinsed in 0.9 % saline for 1 min to remove non-adherent bacteria. The samples were then fixed with 2.5 % glutaraldehyde (Kanto Chemical Co., Inc., Tokyo, Japan) in 0.1 M cacodylic acid (Wako Pure Chemical Industries, Ltd., Miyagi, Japan) at 4 °C for 16 h. The pegs were washed in 0.1 M cacodylic acid and then washed once in distilled water for approximately 10 min. Saturated 70 % ethanol was applied for 15–20 min and then the sample was air dried for a minimum of 24 h. Specimens were finally mounted and examined using FE-SEM.

### EGCG, LL-37 and LTA interaction analysis using quartz crystal microbalance (QCM)

QCM was used to analyze the potential enhancement effect of LL-37 on binding between EGCG and bacterial LTA. EGCG was used as a ligand and LTA from *S. mutans* (L4152; Sigma-Aldrich, St. Louis, MO, USA) was used as an analyst. QCM measurements were performed using AFFINIX QN μ (INITIUM Inc., Kanagawa, Japan). This instrument has a 500-μL cell equipped with a 27-MHz QCM plate at the bottom of the cell, in addition to a stirring bar and temperature control system. Gold-coated quartz crystal sensor surfaces were washed twice by mounting 3:1 mixture of concentrated sulfuric acid and hydrogen peroxide solution for 5 min. An AFFINIX immobilization kit was then used following the manufacturer’s instruction. Briefly, the surfaces of the sensors were coated with carboxylic acid-terminated thiol and carboxylic acids were activated as N-hydroxysuccinimidyl esters as previously described [34]. Activated carboxyl groups reacted with EGCG (0.2 mg/mL). After the binding of EGCG to the sensor, unreacted esters were deactivated using 1 mol ethanolamine solution. The amount of LTA solution (10 μg/mL) and/or LL-37 (80 μg/mL) injected each time was 5 μL each. HBSS was used as a measurement buffer. The stirring speed was set at 1000 rpm, and experiments were conducted at 25 °C. Frequency changes in response to the addition of LTA solution were monitored in real time. As a control, 10 μg/mL of LTA was injected without initially binding EGCG on the sensor.

The article "Human cathelicidin LL-37 enhance the antibiofilm effect of EGCG on Streptococcus mutans" was retracted in 2017. Reasons: copyright claims; concerns about the data.

### Statistical analysis

Data are presented as the means and standard deviations. Significant differences were determined by the *t*-test using Microsoft Excel 2007 (Microsoft Corporation). Values were considered to be statistically significant at *p* < 0.05.

## Results

### Short-term antibacterial effect of EGCG on the growth of *S. mutans*

In growth inhibition tests, MICs of EGCG for *S. mutans* planktonic cells (*n* = 10) ranged from 0.025 to 0.1 mg/mL; MBCs ranged from 0.1 to 0.4 mg/mL (Additional file 1: Table S1). To determine the kinetics of the antimicrobial activity of EGCG, bacterial suspensions were incubated with varying concentrations of EGCG for 3 and 5 h. The percentage of viable bacteria clearly decreased from 64.7 to 4.0 % and 45.3 to 0 % with the treatment of 0.0125–0.2 mg/mL EGCG after incubation for 3 and 5 h, respectively (Fig. 1). These results show EGCG has a short-term bactericidal effect on *S. mutans*.

**Fig. 1:** Short-term killing assays for EGCG against *S. mutans* (*n* = 10). Standardized overnight cultures of *S. mutans* strains (3000 CFU/mL) were seeded in a 96-well microtiter plate with varying concentrations of EGCG and incubated for 3 and 5 h at 37 °C. Data are presented as the mean ± SEM from three independent experiments. *, significant difference compared with untreated control (*p* < 0.05)

### Inhibitory effect of EGCG on biofilm formation in the presence and absence of LL-37

The inhibitory effect of EGCG with or without LL-37 on biofilm formation of *S. mutans* was measured by crystal violet staining of pegs in MBEC assays. The number of biofilm cells on 0.2 mg/mL EGCG with or without 80 μg/mL LL-37-treated pegs were slightly less than untreated pegs at 12 h and showed a significantly decrease after 24- and 36-h incubation (*p* < 0.05) (Fig. 2). Moreover, EGCG treatment with LL-37 resulted in less adherent bacteria than EGCG treatment alone. These results indicate that the inhibitory effect of EGCG on *S. mutans* biofilm formation could be enhanced by the addition of LL-37.

The article "Human cathelicidin LL-37 enhance the antibiofilm effect of EGCG on Streptococcus mutans" was retracted in 2017. Reasons: copyright claims; concerns about the data.

**Fig. 2:** Biofilm inhibition assay. Standardized overnight cultures of *S. mutans* strains (*n* = 10) were grown on MBEC pegs incubated with 0.2 mg/mL EGCG in the presence or absence of 80 μg/mL LL-37 for 12, 24, or 36 h at 37 °C. Adherent cells were then fixed with ethanol, stained with crystal violet, eluted with ethanol, and the absorbance was measured. Data are presented as the mean ± SD from three independent experiments. *, significant difference compared with untreated control (*p* < 0.05)

### Inhibitory effect of EGCG on preformed *S. mutans* biofilms in the presence and absence of LL-37

The dispersion of preformed biofilms treated with EGCG was then evaluated using biofilm susceptibility assays. *Streptococcus mutans* biofilms were grown on MBEC pegs and then exposed to 0.2 mg/mL EGCG with or without the addition of 80 μg/mL LL-37 in fresh media for 3 and 5 h. After removal of the pegs, the number of viabel bacteria that remained on the pegs was determined using quantitative crystal violet staining. Compared with the control group, *S. mutans* preformed biofilms showed sensitivity to 0.2 mg/mL EGCG treatment, with the highest sensitivity to EGCG in the presence of 80 μg/mL LL-37 at 5 h (Fig. 3).

**Fig. 3:** Biofilm susceptibility assays. Standardized overnight cultures of *S. mutans* strains grown on MBEC pegs and incubated overnight at 37 °C to form mature biofilms. The pegs were immersed in wells containing 0.2 mg/mL EGCG in the presence or absence of 80 μg/mL LL-37 for 3 and 5 h to allow the biofilm to disperse from the pegs to the wells below, and the absorbance was measured. Data are presented as the mean ± SD from three independent experiments. *, significant difference compared with untreated control (*p* < 0.05)

### Effect of EGCG on *S. mutans* cell morphology and biofilm formation

FE-SEM was used to observe the effect of EGCG on *S. mutans* cell morphology and preformed biofilms. As shown in Fig. 4a, the surface of 0.2 mg/mL EGCG-treated cells became rough and exhibited broken membranes with leaked cytoplasm, whereas untreated *S. mutans* cells were smooth (Fig. 4b). Microscopic images of *S. mutans* preformed biofilms on MBEC pegs are shown in Fig. 4c–e, and whole-cell images of treated cells are shown in Additional file 2: Figure S1. EGCG-treated samples had decreased numbers of adherent bacteria and cell membranes were rough. Moreover, the antibiofilm activity of EGCG was more effective in the presence of LL-37.

The article "Human cathelicidin LL-37 enhance the antibiofilm effect of EGCG on Streptococcus mutans" was retracted in 2017. Reasons: copyright claims; concerns about the data.

**Fig. 4:** Changes in number of planktonic cells and preformed biofilms following incubation of EGCG with/without LL-37. Representative images of bacterial cells observed by field emission-scanning electron microscope (working distance: 10 mm, field width: 5 μm) are shown. *Streptococcus mutans* suspensions incubated in the presence (**a**) or absence (**b**) of 0.2 mg/mL EGCG for 24 h. *Streptococcus mutans* biofilms on MBEC pegs incubated with 0.2 mg/mL EGCG (**c**), 0.2 mg/mL EGCG, and 80 μg/mL LL-37 (**d**), or BHI medium (**e**) for 24 h. The white arrow indicates the “ring” phenomena around damaged cells

### Intermolecular interactions with LTA

The preceding experiments indicated that EGCG likely binds to a component in the bacterial membrane, and this interaction could be enhanced by LL-37. Therefore, we conducted a QCM analysis to determine the precise interaction(s) between EGCG, LL-37, and LTA. In the control experiment, the frequency decreased to below the significance level. The level of decrease caused by non-specific binding between LTA and the blocking agent was 12 Hz. When 1 mg/mL LTA was added, the frequency decreased by 162 Hz, indicating disruption of the interaction between EGCG and LTA. When 80 μg/mL of LL-37 was added, the frequency decreased by 313 Hz, indicating an intermolecular interaction between EGCG and LL-37. After the addition of 1 mg/mL LTA and 80 μg/mL LL-37, the frequency decreased by 524 Hz. These results suggest that EGCG interacts with LTA through binding of LL-37.

## Discussion

Catechins have a broad spectrum of antimicrobial activity against both Gram-positive and Gram-negative bacteria, especially galloylated derivatives such as EGCG, which have been documented to possess antimicrobial effects against oral streptococci [11]. According to our early study, EGCG demonstrates the highest activity against *S. mutans* [28], which also supported by other researches [20, 21, 31, 35].

Biofilms increase the ability of bacteria to resist most antibiotics and therapeutic agents [36]. Stable biofilm formation is also considered one of the key factors of caries pathogenesis. In this study, the inhibitory effect of EGCG on *S. mutans* planktonic cells, biofilm formation, and mature biofilms was examined. EGCG was found to inhibit visible bacterial growth at 0.1 mg/mL, decrease biofilm formation, and exhibit a bactericidal effect on preformed biofilms at 0.2 mg/mL (data not shown). *Streptococcus mutans* in biofilms displayed lower susceptibility to EGCG compared with planktonic bacteria [20]. We also observed that EGCG treatment reduced attachment of *S. mutans*, as previously shown [21], and caused changes in the cell membrane. Based on these results, the antimicrobial mechanism of EGCG is likely attributable to irreversible damage of the microbial cytoplasmic membrane, as previously described [37].

The article "Human cathelicidin LL-37 enhance the antibiofilm effect of EGCG on Streptococcus mutans" was retracted in 2017. Reasons: copyright claims; concerns about the data.

LL-37, which is expressed in many tissues and body fluids, has a broad spectrum of antimicrobial activity against both Gram-positive and Gram-negative bacteria, including *Staphylococcus aureus* and *Pseudomonas aeruginosa*. In our previous study, we showed that *S. mutans* was resistant to LL-37 in growth inhibition and bactericidal tests, but sensitive to LL-37 during biofilm formation, which was partly because of binding to LTA [28]. In this study, we observed that EGCG had an inhibitory effect on *S. mutans* biofilm formation and reduced the viability of preformed biofilms, without interacting with LTA. Therefore, we analyzed the potential cooperative antibacterial effect of EGCG and LL-37. Our results showed that LL-37 has no effect on the antibacterial effect of EGCG on *S. mutans* planktonic cells (data not shown), whereas it plays an enhancer role in the inhibition ability of EGCG on preformed biofilms. The number of bacteria in preformed biofilms was decreased in the presence of LL-37 compared with EGCG treatment alone, which was confirmed by FE-SEM. This indicates that LL-37 may enhance the antibiofilm effect of EGCG on *S. mutans*.

To understand the LL-37 enhancement effect on the antibiofilm activity of EGCG, we subsequently analyzed the interaction among EGCG, LL-37, and LTA of *S. mutans*. EGCG lacked direct interaction with LTA of *S. mutans*. In our previous study, we demonstrated that LL-37 can interact with LTA on *S. mutans* [28]. In this study, EGCG and LL-37 exhibited a synergistic antibiofilm effect on *S. mutans* (Fig. 5). We hypothesize the two following mechanisms: 1) LL-37 binds to LTA of *S. mutans*, enhancing the attachment site of EGCG; or 2) LL-37 interacts with EGCG, raising the cations on EGCG and increasing the affinity between EGCG and LTA, which is supported by Heptinstall et al. [38]. Further studies on the precise mechanism(s) by which LL-37 enhances the antibiofilm effect of EGCG on *S. mutans* are necessary.

**Fig. 5:** Interaction among EGCG, LL-37, and LTA of *S. mutans*. Graphs show the change in delta frequency after injecting LTA and/or LL-37 on the sensor of quartz crystal microbalance. Five microliters of LTA (1 mg/mL) and/or LL-37 (8 mg/mL) were injected. The final concentrations of LTA and LL-37 were 10 and 80 μg/mL, respectively. LTA without initially binding EGCG was injected on the sensor as a control. Data presented are representative of three independent experiments with similar results

The article "Human cathelicidin LL-37 enhance the antibiofilm effect of EGCG on Streptococcus mutans" was retracted in 2017. Reasons: copyright claims; concerns about the data.

## Conclusions

Our results indicated that LL-37 can enhance the antibiofilm effect of EGCG on *S. mutans* biofilms. This finding provides new knowledge for dental treatment by using LL-37 as a potential antibiofilm compound.

## Additional files

Additional file 1: Table S1. Growth inhibition of *S. mutans*. (DOC 32 kb) Additional file 2: Figure S1. Changes in *S. mutans* preformed biofilms with EGCG treatment with/without LL-37 for 24 h. (PDF 258 kb)

## Abbreviations

BHI: Brain heart infusion
CFU: Colony-forming unit
CLSI: Clinical and laboratory standards institute
EGC: (−)-epigallocatechin
EGCG: (−)-epigallocatechin gallate
FE-SEM: Field emission-scanning electron microscopy
HBSS: Hank’s balanced salt solution
HTP: High-throughput
LL-37: Human cathelidicin
LTA: Lipoteichoic acids
MBC: Minimum bactericidal concentration
MBEC: Minimum biofilm eradication concentration
MIC: Minimum inhibitory concentration
PBS: Phosphate buffered solution
QCM: Quartz crystal microbalance
